# The Application of Natural Camel Milk Products to Treat Autism-Spectrum Disorders: Risk Assessment and Meta-Analysis of Randomized Clinical Trials

This article has been retracted.

**DOI:** 10.1155/2022/6422208

**Published:** 2022-05-27

**Authors:** Mahmoud Kandeel, Wael El-Deeb

**Affiliations:** ^1^Department of Biomedical Sciences, College of Veterinary Medicine, King Faisal University, Al-Hofuf 31982, Al-Ahsa, Saudi Arabia; ^2^Department of Pharmacology, Faculty of Veterinary Medicine, Kafrelshikh University, Kafr El-Shikh 33516, Egypt; ^3^Department of Clinical Sciences, College of Veterinary Medicine, King Faisal University, Al Hofuf, Al-Ahsa, Saudi Arabia; ^4^Department of Internal Medicine,Infectious Diseases and Fish Diseases, Faculty of Veterinary Medicine, Mansoura University, Manosura, Egypt

## Abstract

Camel milk is better tolerated than the milk of other ruminants, potentially expanding its consumer appeal. It also contains essential vitamins, minerals, and immunoglobulins, providing the milk with antioxidant, antibacterial, and antiviral properties. These properties may reduce oxidative stress in camel milk consumers, ameliorating many conditions, including those of the CNS, such as autism spectrum disorders (ASDs). We performed a meta-analysis of randomized controlled trials (RCTs) in which camel milk administration (boiled or raw) was examined as an ASD treatment intervention. The primary endpoint was participants' total autism scores, determined using the Childhood Autistic Responsiveness Scale (CARS). A comparison of the responsiveness in these ASD intervention groups yielded a mean difference (MD) of 1.99 (0.89, 3.08) in those consuming boiled camel milk, MD = 2.77 (1.92, 3.61) in raw camel milk consumers, and MD = −1.02 (−0.10, 2.13) in cow milk consumers. Heterogeneity was notably low among the examined studies. Treatment of ASD with raw and boiled camel milk resulted in significantly lower CARS scores than the placebo. Our findings support the development of larger, more populated RCTs to establish camel milk's overall potential as a therapeutic intervention for CNS disorders.

## 1. Introduction

In many countries, milk has long been a staple component of the human diet. Currently, cow milk production is a significant cause of environmental concern, as it leads to substantial carbon/methane emissions, water pollution, soil erosion, and over-foraging. In contrast to cows, milk-producing camels, primarily reared in the Middle East and North Africa, are considered eco-friendly, low-waste animals [1]. Camels generate less than half the carbon emissions of dairy cows and are more efficient milk producers. Furthermore, their milk is considered more nutritionally beneficial. Recently, camels have been associated with MERS-CoV, an emerging coronavirus [2, 3]. Although there are unresolved questions regarding the zoonotic aspects of MERS-CoV, specific camel milk antibodies may also provide coronavirus cross-protection [4].

Researchers have demonstrated the therapeutic value of camel milk in managing diabetes [5–7], hepatitis B [8], hepatitis C [9], *Helicobacter pylori* infections, enterocolitis, lactase deficiency in children [10, 11], pulmonary tuberculosis [12], liver cirrhosis [13], and cancer [14]. Furthermore, the unique composition of camel milk includes multiple protective proteins such as lysozymes, immunoglobulins, and lactoperoxidase, making it similar to human breast milk and serving to protect against infection and bolster immunological responses [15, 16].

Camel milk is also low in cholesterol, lactose, and fat content [17] and high in vitamins and minerals, most abundantly sodium, magnesium, zinc, copper, and potassium [18]. Specifically, camel milk has higher concentrations of vitamins A, B2, C, and E [19, 20] and higher zinc and iron concentrations than goat or cow milk. Moreover, camel milk contains a relatively high amount of polyunsaturated fats and linoleic and linolenic fatty acids, which are essential for human nutrition [21]. The IgA and IgG immunoglobins in camel milk provide significant protection against viruses and bacteria. Casein is the primary protein found in camel milk, and its association with other whey proteins supplies albumin, immunoglobins, and lactoferrins. Furthermore, lysine, threonine, valine (all essential amino acids) and glycine are predominant in camel milk [22].

Autism spectrum disorder (ASD) is a collection of developmental impairments manifested by challenges in communication and interpersonal interactions, stereotypical behaviors, and limited interactions. Early studies demonstrated that ASDs were significantly heritable [23] and have been observed to exhibit high phenotypic heterogeneity regarding presentation during human development. However, the root cause of ASD remains undetermined and, at times, contentious. A strong association has been found between ASD development and autoimmunity [24], based on the high prevalence of brain-specific autoantibodies in the brains of children with autism. The mechanism of autoantibody development in the brain is still not adequately understood. Some have speculated that they trigger autoimmune reactions in neurons via cross-reactive neuronal antigens [25]. Furthermore, oxidative stress [26, 27] and genetic polymorphism [28] have also been proposed to be involved in ASD pathogenesis. One study revealed that an increased number of neuropeptides in the brain could be responsible for neurogenic inflammation in ASD pathogenesis [29].

The correlation between camel milk consumption and protection against inflammation [30], hepatotoxins, carcinogens [31], diabetic complications, autoimmunity, and multiple sclerosis associated with ASDs [32, 33] has increased the global demand for camel milk products [34]. Multiple studies have examined camel milk as a potential alternative and supplemental therapy for ASDs. To assess this body of work, we performed a meta-analysis of randomized controlled trials (RCTs) on the use of camel milk to treat various CNS conditions. Our results reveal that patients treated with raw or boiled camel milk had lower Childhood Autism Responsiveness Scale (CARS) scores, indicating that camel milk may reduce neuroinflammation or autoimmunological responses associated with ASDs.

## 2. Materials and Methods

### 2.1. Objectives

In accordance with guidelines established by the Preferred Report Items for Systematic Review and Meta-Analysis (PRISMA), a PICO (Population, Intervention, Comparison, and Outcomes) strategy was employed to analyze the contribution of camel milk consumption to reductions in ASD-associated behaviors as measured by CARS.

#### 2.1.1. Population

The meta-analysis included patients diagnosed with autistic spectrum disorders (ASDs).

#### 2.1.2. Intervention

The intervention was the administration of raw or boiled camel milk and cow milk (as a placebo) in ASD patients. CARS scores were measured before, immediately following, and two weeks after administration in all the RCTs included in this meta-analysis.

#### 2.1.3. Benefit Comparison

We compared the benefits associated with camel milk administration in ASD treatment using the following measurements: CARS and vasoactive intestinal peptide (VIP) scores; blood plasma concentrations of myeloperoxidase, superoxide dismutase, and glutathione; serum levels of thymus and activation-regulated chemokines (TARC); and the autism evaluation checklist.

### 2.2. Search Strategy

The Cochrane Database of Systematic Reviews, EMBASE, PubMed, and Web of Science medical databases were searched for RCTs. There was an electronic search for any active clinical trials on the topic. Other potential studies were also found using the Google Scholar search engine. Cited references within the peer-reviewed journal articles were also searched manually.

Keywords indicated the search approach. We extracted literature from 2000 to 2022 using a search method including the English language and chronological filters. The following search terms were used to generate eligible literature: camel milk, CNS diseases, autism, or ASDs.

### 2.3. Eligibility Criteria

#### 2.3.1. Inclusion Criteria

Studies with abstracts and articles included in the meta-analysis met the following inclusion criteria: (1) reported risk estimates, (2) provided novel research results or included RCTs, (3) conducted no earlier than the year 2000, (4) detailed CNS diseases, and (5) reported in the English language.

### 2.4. Study Selection and Data Synthesis

Two researchers conducted a standardized and systematic review of the relevant available data. Each analyzed database was utilized in conjunction with the inclusion criteria to determine if an abstract was included or omitted from consideration. Each researcher selected and reviewed individually the full-length papers that were accepted for consideration. In cases where the primary author's information could not be obtained, the chief researcher validated the discrepancies independently. After reaching a consensus, any conflicts that arose were analyzed and resolved to provide data with the greatest degree of transparency.

### 2.5. Data Analysis

Data derived by a thorough search of the medical databases for eligible criteria were tabulated in the study identification. The country in which each study was conducted and other demographic characteristics of the included studies were included in the analysis. Perceived outcomes from each study were also included in the tabulated file, showing all relevant characteristics of each study.

Since all included studies included data from RCTs, a meta-analysis was conducted using the Cochrane tool for systematic reviews and meta-analysis. An inverse variance weighted random model was utilized to calculate the risk ratio using a 95% confidence interval of dichotomous data and a standard mean difference of continuous data. Heterogeneity was also measured for all expected outcomes, with results of *p* < 0.05 considered statistically significant.

### 2.6. Risk of Bias

The efficacy of an intervention might be underestimated or overstated due to flaws in RCT design, methodology, analysis, and reporting. The technique developed by the Cochrane Collaboration to measure bias risk attempts to make the process more transparent and accurate [35]. To reduce bias, we employed obfuscated randomization, explicit inclusion and exclusion procedures, the blinding of the study, individual screening, blinded data processing, and intention-to-treat analysis. The total risk of bias in the studies was assessed using the Cochrane Handbook Tool for Risk of Bias [35]. The studies were categorized as demonstrating a high, low, or uncertain probability of being biased. Data from sequence construction, allocation concealment, participant, staff, and result assessor blinding, inadequate data, selective outcome reporting, and other risks were included in the overall risk of summary bias (Figure 1).

## 3. Results

We identified 400 eligible published and gray literature studies in several medical databases on the benefits of treating CNS diseases with camel milk. Forty-five studies included animal trial data, 54 were case reports, systematic reviews, and meta-analyses, 60 focused on alternate conditions, and 30 and 70 studies reported only on care and management and nonoral feeding, respectively.

Further stratification of the available literature yielded 24 studies. Careful analysis of the extracted literature resulted in excluding six studies as they were not RCTs. An additional 15 studies were excluded as they focused on other diseases. Finally, four studies were selected for a systematic review and a meta-analysis (Figure 2). A summary of study characteristics, comprising the study ID, design, population, duration, and outcomes, is provided in Table 1. Forest-plot analyses of the results are provided in Figures 3–5.

A comparison of the different levels of responsiveness in these groups revealed a mean difference (MD) of 1.99 (0.89, 3.08) in the ASD intervention group treated with boiled camel milk, MD = [2.77 (1.92, 3.61)] in the ASD intervention group treated with raw camel milk, and MD [1.02 (−0.10, 2.13)] in the cow milk group. The investigated studies demonstrated a low level of heterogeneity. Treatment of ASD with raw and boiled camel milk resulted in significantly lower CARS scores than the placebo.

## 4. Discussion

ASD is now generally recognized as a complex, widespread, heterogeneous syndrome with multiple etiologies, subtypes, and developmental paths. Despite significant social and economic consequences, there are few treatment options for ASD symptoms, which include both diagnostic criteria-related symptoms and those thought to be a result of comorbid mental and medical problems that enhance presentation severity. Researchers have identified camel milk as an effective treatment intervention for ASD in children, especially in the Middle East, where camel milk products are in high demand by consumers. Camel milk may provide an alternative ASD treatment as it is more tolerated than the milk of other ruminants [13]. The results of our meta-analysis highlight the need for broader, more populated RCTs investigating camel milk as an ASD therapeutic.

An analysis of data presented by the included studies in this work shows marginally lower behavioral CARS scores (*p*=0.007) in patients treated with raw or boiled camel milk. This trend is mainly attributed to the ability of camel milk to significantly decrease neuroinflammation and autoimmune reactions [10, 11, 32, 36]. ASD is a life-long condition characterized by an impairment in communication and social interaction [37]. Studies into the causes of ASD have revealed that oxidative stress is a critical risk factor in developing autoimmunity. The vitamin C concentration in camel milk, uniquely higher than other milk products, may be responsible for the antioxidant properties [38]. The availability of many antioxidant vitamins A, C, and E and elevated concentrations of zinc and magnesium minerals in camel milk justifies its use as an antioxidant intervention in ASD patients [19]. Camel milk is also unique in its glutathione and antioxidant mineral concentrations. In the studies included in our meta-analysis, increased blood plasma glutathione, superoxide dismutase, and myeloperoxidase concentrations were observed in ASD patients after consuming camel milk for two weeks. These observations demonstrate the overall therapeutic potential of camel milk consumption due to the reduction of oxidative stress via changes in the concentrations of antioxidative enzymes and nonenzymatic antioxidant molecules [39].

Camel milk has a different casein protein distribution than cow milk, with a lower proportion of A1 *β*-casein. This casein breaks down into its peptide components, including BCM-7, an active opioid that may seep through a person's “leaky gut” and reach the brain, potentially impairing social interaction in ASD patients [40, 41].

Adams (2013) presented a case report on the efficacy of camel milk for the treatment of ASD in children [42]. After consuming camel milk, the patient displayed a significant improvement in the phenotypic ASD manifestations. These changes were highlighted by an “improvement in eye contact, communication, emotional expressions, and self-organization.” Notably, after consuming camel milk for three weeks, the patient exhibited significant improvements in behavior modification, motor function, language, and academic skills and planning, a decreased irritability score and erratic behavior, and improved skin condition. Furthermore, interruptions in camel milk intake resulted in behavioral and physiological impairments and the patient's return to erratic behavior, which decreased when camel milk consumption was resumed.

The strong association between ASD and gastrointestinal difficulties, as manifested in most individuals with ASD, challenges the effective digestion of most milk protein as presented in cow (but not camel) milk. The form of milk protein casein and IgG and IgA immunoglobulins in camel milk also contribute to its potential in ASD intervention. As the immunoglobulins present in camel milk are smaller, they can more effectively penetrate tissues and cells than larger cow milk immunoglobulins [43].

### 4.1. Strengths and Limitations

This meta-analysis assessed the growing and sometimes conflicting data on the influence of camel milk on ASD. We faced several challenges in drafting a full systematic review and meta-analysis. First, research on camel milk treatment of CNS diseases such as ASD is a new field of study. Knowledge of its treatment potential may only be available where camels are abundant, such as in the Middle East, North Africa, and some parts of West and East Africa. This limitation resulted in a very small number of RCTs available for inclusion in this meta-analysis.

Secondly, most of the included studies utilized short treatment time frames, none exceeding two weeks. This observation poses the question of whether the potential benefits of camel milk as an intervention measure for CNS diseases would be observed over the long term. Finally, the conflicting results in the CARS scores presented in the most recent study in 2021 [36] illustrate the need for research investigating the role of camel milk as an intervention for CNS conditions.

## 5. Conclusions

The findings of this study indicate that several critical components of camel milk may help improve ASD symptoms and the autistic patient's quality of life. The unique composition of camel milk, including protective proteins, vitamins, essential mineral ions such as zinc and magnesium, and small immunoglobulins, similar to those found in human breast milk, is a major factor in its growing popularity as a treatment intervention for a variety of conditions. However, evidence from RCTs emphasizing the possible advantages of camel milk consumption remains sparse. Consequently, we propose that longer, more populated RCTs are needed to evaluate these potential benefits. Results derived from the systematic review and meta-analysis highlight some essential components of camel milk aimed at improving ASD diseases and the quality of life of an autistic individual. The unique composition of camel milk with protective proteins, vitamins, essential nutritional mineral ions such as zinc and magnesium, and small immunoglobulins, similar to those found in human breast milk is a major contributing factor to the rise in popularity of camel milk as a treatment intervention for a number of diseases. However, data from randomized clinical trials highlighting the potential benefits remain limited; thus, we advocate for longer, more populated RCTs to carefully examine these benefits.

## Figures and Tables

**Figure 1:** The risk of summary biases reported in the RCTs.

**Figure 2:** Flowchart of the literature search process and results.

**Figure 3:** Forest plot of the meta-analysis results showing the effects of treatment on ASD patients consuming raw camel milk.

**Figure 4:** Forest plot of the meta-analysis results showing the effects of treatment on ASD patients consuming boiled/pasteurized camel milk.

**Figure 5:** Forest plot of the meta-analysis results showing the effects of treatment on ASD patients consuming cow milk (placebo).

**Table 1:** Characteristics of studies included in the meta-analysis of the effects of camel milk consumption on CNS symptoms.

Study ID	Design	Population	Duration	Outcomes
Al-Ayadhi et al. [11]	Double-blinded randomized controlled trial (RCT)	*N* = 65 children with ASD administration of raw camel milk: *n* = 22 boiled camel milk: *n* = 25 placebo: *n* = 18	Two weeks	The study measured the overall rating of the intervention group using the childhood autism rating scale (CARS), the social responsiveness scale (SRS), and the autism evaluation checklist (ATEC). Significant CARS score changes were detected in the intervention groups administered raw and boiled camel milk, and no changes were detected in the placebo group administered cow milk. Social cognition, communication, and awareness were significantly improved in the raw and boiled camel milk treatment groups. This trend was not replicated in the placebo group treated with cow milk. However, the ATEC scores were not significantly different between the three intervention groups. A slight improvement was observed in the speech/communication field in children treated with boiled camel milk.

Mostafa et al. [36]	RCT	*N* = 65 children with ASD administration of raw camel milk: *n* = 24 boiled camel milk: *n* = 23 placebo: *n* = 18	Two weeks	CARS and serum vasoactive intestinal peptide (VIP) scores were measured before and immediately after consuming 500 mL of camel milk in the three intervention groups. An increased VIP mean serum value score was determined after participants consumed boiled camel milk. The CARS scores slightly decreased, and VIP scores increased during treatment with raw camel milk. However, the lack of statistical significance indicated that additional studies conducted over a longer period were needed.

Bashir and Al-Ayadhi [10]	Double-blinded, placebo-controlled trial	*N* = 45 administration of raw camel milk: *n* = 15 boiled camel milk: *n* = 15 placebo: *n* = 15	Two weeks	The primary studied outcomes were the thymus and activation-regulated chemokine (TARC) concentrations and CARS scores. A significant decrease in TARC levels in the blood samples of children consuming raw and boiled camel milk was identified after a two-week intervention. No changes were observed in the placebo group. A significant CARS score difference was only observed in the raw camel milk treatment group.

Al-Ayadhi et al. [32]	Double-blinded RCT	*N* = 60 ASD patients administration of raw camel milk: *n* = 24 boiled camel milk: *n* = 25 placebo: *n* = 11	Two weeks	The overarching objective of the trial was to assess the role of camel milk on oxidative stress exhibited by ASD patients via measurements of the blood plasma levels of glutathione, superoxide dismutase, and myeloperoxidase. Significantly higher glutathione blood plasma levels were observed in the group consuming raw milk and the boiled camel milk-controlled group but not in the placebo group. Furthermore, superoxide dismutase was significantly increased in the raw and boiled camel milk group treatments.

## Data Availability

The data used to support the findings of this study are included within the article.
